RETRACTED

# WELL.ME - Wellbeing therapy based on real-time personalized mobile architecture, *vs.* cognitive therapy, to reduce psychological distress and promote healthy lifestyle in cardiovascular disease patients: study protocol for a randomized controlled trial

**DOI:** 10.1186/1745-6215-13-157

**Published:** 2012-09-03

**Authors:** Angelo Compare, Vassilis Kouloulias, Vontas Apostolos, Wendy Moreno Peña, Enrico Molinari, Enzo Grossi, Efstathopoulos Efstathios, Michele Carenini

**Affiliations:** 1 Human Factors and Technologies for Health - HTC Centre; Dept. of Human and Social Sciences, University of Bergamo, Piazzale S. Agostino 2, 24129, Bergamo, BG, Italy; 2 Medical School, National University of Athens, Athens, Greece; 3 Technopolis ICT Business Park, Thessaloniki, Greece; 4 SOROS GABINETE, Socia ProgramasEuropeos, Europe, Spain; 5 Istituto Auxologico Italiano; Catholic University of Milan, Milan, Italy; 6 Medical Department, Bracco SpA; IULM - University, Fondazione Bracco, Milan, Italy; 7 NoemaLife Spa, Bologna, Italy

**Keywords:** Anxiety, Depression, Psychological distress, Cognitive behavior therapy, Wellbeing therapy, Mobile technology, Cardiac disease

## Abstract

**Background:**

There is compelling evidence that psychological factors may have the same or even greater impact on the possibility of adverse events on cardiac diseases (CD) than other traditional clinical risk factors. Anxiety and depression are predictors of short- and long-term adverse outcomes, increased risk for higher rates of in-hospital complications, re-infarction, malignant arrhythmias, and mortality in CD patients. Despite researchers finding that cognitive behavior therapy (CBT) reduced depressive and anxiety symptoms, the fact that such results are maintained only in the short term and the lack of maintenance of the long-term affects the absence of changes in lifestyles, preventing the possibility of a wide generalization of results. Recently wellbeing therapy (WBT) has been proposed as a useful approach to improve healthy lifestyle behaviors and reduce psychological distress.

**Methods/design:**

The present randomized controlled study will test WBT, in comparison with CBT, as far as the reduction of symptoms of depression, anxiety and psychological distress, and the improvement of lifestyle behaviors and quality of life in cardiac patients are concerned. Moreover, innovations in communication technologies allow patients to be constantly followed in real life. Therefore WBT based on personalized mobile technology will allow the testing of its effectiveness in comparison with usual WBT.

**Discussion:**

The present study is a large outpatient study on the treatment of co-morbid depression, anxiety, and psychological distress in cardiac patients. The most important issues of this study are its randomized design, the focus on promotion of health-related behaviors, and the use of innovative technologies supporting patients’ wellbeing in real life and in a continuous way. First results are expected in 2012.

RETRACTED

**Trial registration:**

ClinicalTrials.gov Identifier: NCT01543815.

## Background

Cardiac disease (CD) is the major cause of death worldwide, accounting for approximately 16.7 million deaths each year, mainly from heart attack and stroke. Furthermore, such a figure is most likely to increase approximately to 25 million deaths by 2020, given current trends. Yet fatalities represent only the tip of the iceberg; the greater burden of cardiovascular diseases, affecting an estimated 128 million people, is attributable to non-fatal cardiovascular events and their long-term consequences. Although there are well-accepted national guidelines for both primary and secondary prevention of cardiac illness, little attention has been devoted to the impact of psychological risk factors on cardiovascular disease. Nonetheless, there is wide evidence that psychological risk factors may cause equal or even more adverse events than other traditional clinical risk factors [1-4].

In patients with ischemic heart disease, anxiety and depression are predictors of adverse short- and long-term outcomes [5,6]. Patients suffering from anxiety or depression during hospital admission are at increased risk for higher rates of in-hospital complications such as recurrent ischemia, re-infarction, and malignant arrhythmias [7,8]. They also suffer higher mortality and re-infarction rates months to years after their initial cardiac event [8-11].

Affective disorders including clinical depression and anxiety are common in patients with congestive heart failure. Prevalence findings show that the prevalence rates of (all subtypes) anxiety and depression are 18.4% and 28.6%, respectively [12], and depression is a significant predictor of worse evolution for heart failure (HF) patients [13]. Furthermore, the occurrence of such disorders significantly impacts the quality of life, medical outcomes, and the use of the healthcare service. A number of potential mechanisms have been proposed to justify such an impact, including autonomic nervous system dysfunction, inflammation, cardiac arrhythmias, and altered platelet function.

The relationship between emotional distress and the experience of fatigue in patients with HF may have a devastating effect on a patient’s ability to cope with and manage daily activities, including self-care and adherence to recommended treatment. Reports show that anxiety is associated with mental fatigue, whereas depression is associated with the reduction of activity, low motivation, and the assumption of lifestyles which are dysfunctional towards a healthy status. Moreover physical fatigue is affected by symptomatic distress [14].

RETRACTED

In everyday practice it is important to consider that a high NYHA classification together with emotional problems may contribute to anxiety or depression, while social support and active relationships may positively influence the psychological health of patients with heart failure [15]. In particular, baseline distress assessed in primary care (odds ratios (OR) 5.51; 95% confidence intervals (CI) = 2.56 to 11.62) appears to be an independent predictor of distress at 9-monthfollow-up. Recent findings show that anxiety and low social support were independently associated with HF-related re-admission, which indicates the need for their inclusion in the assessment and management of HF [16]. Moreover, data show that depression ((HR = 1.81) and social isolation (HR = 2.25) may be mortality predictors independently of demographics, clinical predictors, and treatment [17].

Failure to understand and address psychological risk factors for coronary heart disease(CHD) events may be one reason for which CHD morbidity and mortality remain so high. Anxiety disorders and depression are among the most prevalent psychiatric disorders [18]. Given the prevalence of anxiety and depression in the general population and in patients with CHD, the potential public health impact for preventing the development and progression of CHD by properly appreciating the nature of the link between anxiety or depression and CHD is enormous [19,20]. Thus, in CVD patients it is clinically relevant to assess the patient’s psychological profile and treat his/her emotional conditions causing an increased risk for major adverse cardiovascular events.

### Psychological interventions for anxiety and depression

Major behavioral and drug trials conducted in the last 15 years have focused on the best treatment of depression in cardiac patients [21]. Cognitive behavioral therapy (CBT) is often successfully used in the treatment of depressive disorders. Although the adoption of CBT obtained good results in reducing depression, no beneficial effects for cardiac events in 2 years was reached inpatients receiving the intervention (24.2%) when compared with a control group undergoing a usual treatment (24.1%). Because dysfunctional cognition plays a relatively minor role in atypical depression, treatments other than cognitive-behavioral interventions may be more beneficial to CHD patients with atypical depression or exhaustion [22]. Moreover, CBT is a well-documented, evidence-based treatment appropriate for the treatment of anxiety, which should be started at the beginning of cardiac treatment to ensure that patients fully understand their condition [23].

RETRACTED

Despite researchers finding that CBT reduces depressive and anxiety symptoms, the limited size of studies prevents a wide generalization of the results [24].

Recently wellbeing therapy (WBT) has been proposed as a useful approach to improve healthy lifestyle behaviors and reduce psychological distress. WBT aims at enhancing psychological wellbeing on the basis of Ryff’s [25] six dimensions: autonomy, personal growth, environmental mastery, purpose in life, positive relations, and self-acceptance. Previous studies documented the efficacy of this psychotherapy in treating patients with mood and anxiety disorders, and in preventing relapse in recurrent depression [26-28]. Moreover, recent results showed that a sequential combination of CBT and WBT yield significant and persistent benefits in cyclothymic disorder [29].

## Methods/Design

### Hypotheses

Starting from current literature, we hypothesize that WBT and WBT version based on a personalized mobile technology approach will allow for a reduction of symptoms of depression, anxiety, and psychological distress in cardiac patients. Moreover and therefore, we assume an improvement in lifestyle behaviors (for example, quitting smoke, increased physical activity, better medication adherence) and quality of life when compared to CBT and usual care (UC).

### Setting

The study will be conducted in collaboration with the National Kapodistrian University of Athens, Greece, and Consorci Sanitari de Terrassa (CST), Spain, during the 3-year EU collaboration project FOR ALL (‘Universal Service for Managing and Monitoring Cardiac and Psychological Health of European Cardiac Patients’, Project No. C-029399).

### Subjects

Patients with the following eligibility criteria have been included in the present study: cardiac disease; a current diagnosis of at least one of the following: major or minor depression, dysthymia, anxiety according to DSM-IV criteria and HADS criteria, Mini-Mental State Examination score higher than 24;written informed consent was requested from the patient. Exclusion criteria included: uncertain prognosis for 12 months due to other conditions; acute coronary disease in the last 2 months; existence of another life-threatening illness of the patient (such as active cancer, chronic kidney failure); severe neurological problem (brain syndrome/orientation problem/difficult peripheral neuropathy); severe mental illness (active psychosis/suicide risk/severe dementia); linguistic limitations (such as stuttering/untreated audio impairment); a significant functional problem (such as unconsciousness/connection to respiration device/confinement to a wheelchair or bed/severe walking disability/need of help with basic daily activities); objective limit endangering liability for participation in the seven meetings (such as remote living location/convict/drug addiction).

RETRACTED

All eligible patients will be approached by trained clinical psychologists during their hospitalization period and will be screened for depression, anxiety, and psychological distress (Screening phase). Patients with elevated scores on such scales will be invited for a baseline interview to further identify possible exclusion criteria. After this interview, patients satisfying inclusion criteria are further informed about the design of the study and asked to give their informed consent (Evaluation phase). Informed consent will be sought for:(a) using anonymous data from the questionnaires for reports and scientific publications; and (b) for informing the general practitioner (GP) about the study results. Patients will be eventually included in the study and randomized (Randomization phase) to WBT, or WBT-personalized mobile technology platform (MobWBT), either CBT or the care as UC. The phases of the recruitment process are described in Figure 1.

**Figure 1:** **Schematic outline of flow chart of WELL.ME study.** During the Screening phase, patients with high anxiety, depression, and psychological distress will be detected. At Evaluation, inclusion and exclusion criteria will be assessed. After this, the first randomization in three arms (CBT, WBT, and CU)will be done. After the 7 weeks of treatment, the second randomization will be done in WBT arms, obtaining two sub-arms: WBT and MobWBT.

### Randomization

Randomization will be performed by statistical experts of the team study using a computerized random number generator at http:// http://www.randomization.com. Randomization will occur after the baseline measurements and, only in WBT group, after the first randomization (Figure 1). To obtain equal numbers in both conditions, a block randomization design is chosen. After the completion of the inclusion procedure, the clinical psychologist will obtain the file containing the condition to which the patient is allocated.

### Design

The comparison among WBT, CBT, and CU will be assessed in a three-arm randomized controlled clinical trial. After this first randomization, patients in WBT group will be randomized across WBT and MobWBT.

### Intervention

#### Wellbeing therapy (WBT) and WBT based on mobile technology tool (MobWBT)

WBT is based on Ryff’s cognitive model of psychological wellbeing [25]. This model was selected on the basis of its easy applicability to clinical populations [28]. WBT is divided into three phases (Table 1). 

RETRACTED

**Table 1:** Wellbeing therapy protocol for conventional format (outpatients based tools) and for real-time personalized mobile technologies (Mobile Technology Tool)

**Phases**	**Focus**	**Objectives**	**Outpatient-based tool**	**Mobile technology tool**
Initial phase	Identifying and setting episodes of wellbeing into situational context	Report the circumstances surrounding the episodes of wellbeing rated on a scale of 0 to 100, with zero being absence of wellbeing and 100 being the most intense wellbeing	Diary	Mobile diary, personalized by the baseline assessment results and by an adaptive learning algorithm depending on patient’s answers during mobile monitoring
				Visual analogical scale for wellbeing
				Assessment
		Monitor the quality of experience associated with daily situations (work, leisure, and so on)		
		Identification of instances of wellbeing and of optimal experiences		
Intermediatephase	Remove the obstacles to sustained psychological wellbeing on self-monitoring of moments and feelings of wellbeing and graded task assignments	Identify thoughts and beliefs	Graded task assignments of undertaking particular pleasurable activities for a certain time each day	Electronic personalized task assignment by the baseline assessment results and by an adaptive learning algorithm depending on patient’s answers during mobile monitoring
		Leading to premature interruption of wellbeing		
				Visual analogical scale for wellbeing
				Assessment
		Identify the areas of psychological wellbeing which are unaffected by irrational or automatic thoughts and which are saturated with them		
		Reinforce and encourage activities that are likely to elicit wellbeing and optimal experiences		
Final phase	Be able to readily identify moments of wellbeing	Dimensions of psychological wellbeing are progressively introduced	Graded task assignments of undertaking particular pleasurable activities for a certain time each day	Mobile diary, personalized by the baseline assessment results and by an adaptive learning algorithm depending on patient’s answers during mobile monitoring
	Be aware of interruptions to wellbeing feelings (cognitions)			
		Guide the patient from an impaired level to an optimal level according to the above six dimensions		Electronic personalized task assignment by the baseline assessment results and by an adaptive learning algorithm depending on patient’s answers during mobile monitoring
	Follow optimal experiences			
	Meeting the challenge that may entail optimal experiences is emphasized			
				Visual analogical scale for wellbeing
				Assessment

After the first 7 weeks, patients in the WBT arm will be randomized into two arms: WBT and MobWBT. Patients in the WBT group will not receive any treatments, while patients in MobWBT will be followed by a WBT-Mobile technology tool for 8 weeks (Table 1). Figure 2 shows the MobWBT technology platform. The MobWBT technology platform is based on an elaboration of datasets collected from psychological monitoring in real time and used to train a machine learning algorithm to recognize psychological wellbeing conditions. The algorithm is downloaded onto the smartphone and the training and testing process will be repeated to improve its predictive ability. The final aim of MobWBT technology platform is to identify in realtime the psychological wellbeing condition and deliver personalized WBT techniques precisely at the moment of greatest need.

RETRACTED

**Figure 2:** Wellbeing therapy based on real-time personalized mobile technologies.

#### Cognitive behavioral therapy (CBT)

CBT techniques for anxiety and depression will be performed [30] using a manual protocol.

CBT-Depression is based on cognitive restructuring and behavioral techniques. Such techniques towards curing depression focus on the identification of specific problems linked to behavior and thinking moods. The therapist uses structured learning techniquesto teach patients how to monitor and write down their negative thoughts and mental images. The goal is to recognize how those ideas affect the patients’ mood, behavior, and physical condition. Therapists also teach important coping skills, such as problem solving and planning pleasurable experiences.

CBT-Anxiety addresses negative patterns and distortions in the way we look at the world and at ourselves. The goal of cognitive behavioral therapy for anxiety is to identify and correct these negative thoughts and beliefs. The process involves three steps: Identifying negative thoughts, challenging negative thoughts, replacing negative thoughts with realistic thoughts.

#### Usual care (UC)

In UC no extra intervention is provided. Patients receive care as defined in the usual management program (six annual visits with primary care nurse and cardiologist to monitor disease progression). Patients will be screened througha set of questionnaires to assess depression and anxiety every 2 months to record their psychological symptoms. If scores on these questionnaires indicate a moderate to severe level, a notification is sent to theirGP. However, when necessary patients may always consult their GP and receive treatment for depression/anxiety by the GP, or (after a referral) by a mental health specialist.

RETRACTED

### Treatment procedures

Both WBT and CBT will be conducted for eight 45 minutes sessions. The first two sessions will be conducted in the same week. The remaining six sessions will be conducted over a period of 6 weeks (one session per week). The total therapy duration for each patient will be 7 weeks. Psychotherapy will be provided by clinical psychologists and psychiatrists trained on specific well-assessed treatment protocol.

The Medical Ethics Committee of National Kapodistrian University of Athens and the Consorci Sanitari de Terrassa (CST) approved the study protocol and informed consent. Psychotherapy will be provided individually twice a week.

### Measurements

Besides the psychological screening baseline at month 1 (T_0_), all patients will be assessed at months 6 (T_1_), 12 (T_2_) and 24 (T_3_) for follow-up. Table 2 shows an overview of variables measured at each time point. Moreover, at the baseline assessment, questions on demographic variables (for example, age, marital status, work, educational level, socioeconomic status), psychiatric history (for example, previous diagnosis of depression and/or anxiety, family history regarding psychiatric diagnosis), and/or health behaviors (for example, alcohol use, smoking habits, physical activity) will be included. Clinical variables and diagnosis of other chronic diseases will be obtained from medical records.

**Table 2:** Variables measured at each time point

	**PHQ-9**	**GAD-7**	**DCPR**	**PSI**	**SF-12**	**PGWBI**	**LHFQ**
T_0_	X	X	X	X	X	X	X
T_1_	X	X	X	X			
T_2_	X	X	X	X	X	X	X
T_3_	X	X	X	X	X	X	X

### Primary outcome measures

#### Healthy lifestyle

Diet, physical activity, weight, blood lipids, glucose, and insulin were measured at baseline and at months 6, 12, and 24.

#### Depression and anxiety

The Patient Health Questionnaire-9 (PHQ-9) is a short self-report questionnaire based on the nine symptoms of major depression, as defined in the Diagnostic and Statistical Manual (DSM-IV). The scale has a good overall accuracy, sensitivity, and specificity in a general primary care population [31]. A cutoff of 7can be used to indicate possible depression [32].

The Generalized Anxiety Disorder-7 scale (GAD-7)has shown good reliability and validity to detect generalized anxiety disorder as well as other anxiety disorders in primary care patients [33]. A score >7can be used to indicate a possible anxiety disorder.

The Diagnostic Criteria for Psychosomatic Research (DCPR) [34] represents a diagnostic and conceptual framework that aims at translating psychosocial variables derived from psychosomatic research into operational tools. A set of 12syndromes was developed: disease phobia, thanatophobia, health anxiety, illness denial, persistent somatization, functional somatic symptoms after a psychiatric disorder, conversion symptoms, anniversary reaction, irritable mood, type A behavior, demoralization, and alexithymia.

RETRACTED

The Psychosocial Index (PSI) [35] is a simple self-rated instrument including 55 items for assessing stress, psychological distress, abnormal illness behavior, and wellbeing.

Psychological Wellbeing Scale (PWB) [25] is used in the original 20-item per scale version devised to evaluate six dimensions of well-being: (1) autonomy; (2) environmental mastery; (3) personal growth; (4) positive relationships with others; (5) purpose in life; and (6) self-acceptance.

#### Quality of life/Health status

Health Survey (SF-12) is a health status questionnaire composed by two components (mental and physical) measuring functional status, wellbeing, and general health; higher scores indicate a better health status [36]. The scale was developed to be used in a variety of chronic diseases [37].

The Psychological General Wellbeing Index (PGWBI**)**is an index to measure the level of subjective psychological wellbeing that has been validated by decades of clinical practice. PGWBI has been developed as a tool to measure self-representations of intra-personal affective or emotional states reflecting a sense of subjective wellbeing or distress, thus capturing what we could call a subjective perception of wellbeing [38,39]. The original PGWBI consists of 22 self-administered items, rated on a six-point scale, which assess psychological and general wellbeing of respondents in six health-related quality of life (HRQoL) domains: anxiety; depressed mood; positive wellbeing; self-control; general health; and vitality. Each item may score 0 to 5, referring to the last 4weeks of the subject’s lifetime. Each domain is defined by a minimum of three to a maximum of five items. The scores for all domains can be summarized into a global summary score, which reaches a theoretical maximum of 110 points, representing the best achievable level of wellbeing [38], a sort of ‘state of bliss’. A number of studies are cross-sectional and longitudinal psychometric validation and correlation with a large number of other indexes of medical and mental health, through different contexts (communities, institutions, hospitals) [40]. The average PGWB total score of results from studies of the population is between 80 and 81 points.

Minnesota Living With Heart Failure Questionnaire (LHFQ) [41] measures patients’ perception of the effects of HF in their lives. It is a questionnaire initially prepared to be self-administered, formed by 21 items that contemplate the physical, socioeconomic, and psychological limitations frequently reported by patients connected with their HF. Patients’ self- assessment is quantified by the sum of answers of the 21 items. The scale of answers for each question ranges from 0(‘no’) to 5(‘too many’), where0represents ‘no limitations’ and 5 represents ‘maximum limitation’. Higher scores indicate worse HRQOL.

RETRACTED

### Ethical principles

The study of this protocol does not involve the administration of drugs. However, the investigator is responsible for ensuring that the study is conducted in accordance with the principles defined by the 18th World Medical Assembly (Helsinki, 1964) and subsequent amendments established by the 29th (Tokyo, 1975), 35th (Venice, 1983), 41st (Hong Kong, 1989), and the 48th World Medical Assembly (Somerset West, South Africa, 1996), and 52nd (Edinburgh, Scotland, 2000) General Assembly. The study will also be conducted in accordance to the Ministerial Decree of 15 July 1997 transposing the text of the rules of Good Clinical Practice for human trials of medical products within the EEC.

### Planned statistical analyses

The demographic and clinical characteristics of the two study groups will be compared at baseline to verify their homogeneity. To do this analysis of variance (ANOVA) for continuous variables and chi-square test of Mantel-Haenszel test for discrete variables will be used.

Completer and intent-to-treat analysis will be accomplished to compare treatments both in primary and secondary outcomes. First prevalence of depression, anxiety, and psychological distress will be displayed in frequency tables and both conditions (control and intervention) will be compared using the chi-square (Fisher’s exact test when appropriate) and Student’s t-test, for discrete and continues variables respectively. The effect of the intervention will be determined using multilevel analyses (mixed effect regression models) to compare baseline and follow-up measures of all continuous data. In all these analyses a *P* value of <0.05 will be considered statistically significant.

### Sample size calculation

In this study the change in scores inPHQ-9 and GAD-7 are chosen as primary outcome measures to determine the effect of a disease management approach. A difference of 0.5 standard deviations is considered necessary to find a clinically significant effect of the intervention. In order to detect this difference and assuming a 80% power, a minimum of 80 patients is needed in each condition [42]. When assuming that 20% of participants dropout, quite a normal figure in this type of research, a minimum of 80 patients per condition is needed to maintain sufficient power. We expect that in order to reach such a number, anticipating a response rate of 70% of which 20% is eligible, a total of 600 patients will have to be screened.

RETRACTED

## Discussion

This article describes the background, objectives, and design of a large randomized controlled trial that will test the effectiveness of WBT to treat depression, anxiety, psychological distress, and to improve healthy lifestyle in cardiac disease patients in comparison with CBT and CU. Moreover, the research protocol will test the effectiveness of MobWBT in comparison with WBT. Previous research on cardiac patients has already shown that depression and anxiety are common co-morbidities in these patient populations, and are negatively associated with healthy lifestyle and health status, and positively with morbidity, mortality, and healthcare costs [8-11,17,18]. However, randomized studies on the effects of treating depression, anxiety, and psychological distress are very limited, thus preventing the wide generalization of results [24]. Recently WBT has been proposed as a useful approach to improve healthy lifestyle behaviors and reduce psychological distress. Therefore, this study was developed to test the effectiveness of a WBT approach for co-morbid depression and anxiety in these patient populations. Moreover, innovations in communication technologies allow patients to be followed continuously in real life. Therefore, through WBT based on personalized mobile technology it will be possible to test the effectiveness of these technologies in comparison with usual WBT.

## Conclusions

In conclusion, both depression and anxiety are common diseases in cardiac patients that may provoke a considerable worsening of the cardiac pathology condition. However, research of possible treatment strategies to alleviate this additional burden is limited. Therefore, the WELL.ME study tests the use of WBT to treat co-morbid depression and anxiety in patients with cardiac disease.

## Trial status

The WELL.ME study trial was conceived and designed in 2007. At the time this manuscript was submitted full approval by the Medical Ethics Committee had been obtained.

## Abbreviations

CBT: Cognitive behavioral therapy; CD: Cardiac disease; CHD: Coronary heart disease; CI: Confidence interval; CSM-IV: Diagnostic and Statistical Manual, 4th edition; DCPR: Diagnostic Criteria for Psychosomatic Research; GAD-7: Generalized Anxiety Disorder 7; GP: General practitioner; HF: Heart failure; HRQoL: Health-related quality of life; M.I.N.I.: Mini International Neuropsychiatric Interview; MobWBT: WBT version based on personalized mobile technology; NYHA: New York Heart association; PGWBI: Psychological General Wellbeing Index; LHFQ: Minnesota Living with Heart Failure Questionnaire; OR: Odds ratio; PHQ-9: Patient Health Questionnaire 9; PSI: Psychosocial Index; PWB: Psychological Wellbeing Scale; SPSS: Statistical Package for Social Sciences; UC: Usual care; WBT: Well-being therapy.

RETRACTED

## Competing interests

The authors declare that they have no competing interests.

## Authors’ contributions

AC and VK in collaboration with VA and MC designed the study. All authors have been involved in writing this manuscript and have approved the final manuscript and its submission.

## Funding

EU - eTen Program Grant 2007.
